# Coffee component hydroxyl hydroquinone (HHQ) as a putative ligand for PPAR gamma and implications in breast cancer

**DOI:** 10.1186/1471-2164-14-S5-S6

**Published:** 2013-10-16

**Authors:** Babita Shashni, Karun Sharma, Rumani Singh, Kishore R Sakharkar, Sarinder K Dhillon, Yukio Nagasaki, Meena K Sakharkar

**Affiliations:** 1 Graduate School of Life and Environmental Sciences, University of Tsukuba, Tsukuba, Ibaraki, Japan; 2 AIST, Tsukuba, Japan; 3 OmicsVista, Singapore; 4 Institute of Biological Sciences, Faculty of Science, University Malaya, Kuala Lumpur, Malaysia; 5 Department of Materials Sciences, Graduate School of Pure and Applied Sciences, University of Tsukuba, Ibaraki, Japan; 6 Master's School of Medical Sciences, Graduate School of Comprehensive Human Sciences, University of Tsukuba, Ibaraki, Japan; 7 Satellite Laboratory, International Center for Materials Nanoarchitectonics (WPI-MANA), National Institute for Materials Science (NIMS), University of Tsukuba, Ibaraki, Japan; 8 Department of Biotechnology, University of Pune, Pune, India; 9 Drug Discovery and Development Research Group, College of Pharmacy and Nutrition, University of Saskatchewan, Saskatoon, Canada

## Abstract

**Background:**

Coffee contains several compounds that have the potential to influence breast cancer risk and survival. However, epidemiologic data on the relation between coffee compounds and breast cancer survival are sparse and inconsistent.

**Results:**

We show that coffee component HHQ has significant apoptotic effect on MDA-MB-231 and MCF-7 cells *in vitro*, and that ROS generation, change in mitochondrial membrane permeability, upregulation of Bax and Caspase-8 as well as down regulation of PGK1 and PKM2 expression may be important apoptosis-inducing mechanisms. The results suggest that PPARγ ligands may serve as potential therapeutic agents for breast cancer therapy. HHQ was also validated as a ligand for PPARγ by docking procedure.

**Conclusion:**

This is the first report on the anti-breast cancer (*in vitro*) activity of HHQ.

## Background

Breast cancer is the fifth most common cancer globally and accounts for the highest morbidity and mortality. It is the second highest occurring cancer in women and one of the leading causes of death [1]. Although anti-estrogens have provided an effective endocrine therapy, a significant proportion of patients have acquired resistance to these drugs. Hence, there is a requirement for alternative therapeutics to treat breast cancer. Since, cancer cells modify several pathways to achieve continuous progression and survival, and undergo metabolic alterations, it is important that multiple target strategies are used to achieve effective treatment. Several drugs that inhibit metabolism of cancer cells by targeting a variety of molecules (including enzymes) directly or indirectly are currently under clinical trials, hence it is important to screen drugs with a potential to target critical molecules involved in metabolic transformation [2].

PPARγ receptor is a member of the nuclear receptor superfamily which upon ligand activation undergoes heterodimerization with retinoic acid-like receptor (RXR) and is translocated to the nucleus where it recognizes a specific sequence - the peroxisome proliferator response element (PPRE) located within promoters of target genes, and acts as a transcription regulator for genes involved in proliferation, cell differentiation, apoptosis, angiogenesis, inflammation, organogenesis, and lipid and carbohydrate metabolism and energy homeostasis [3-5]. Two isoforms of PPARγ have been identified (PPARγ 1 and PPARγ 2), with a wide tissue distribution among various animal species [6]. PPARγ are expressed in a variety of tumor cells and PPARγ agonists e.g Thiazolidinediones (TZDs), and tyrosine based agonists show cytostatic and cytotoxic activity against tumor cells *in vitro *and *in vivo *brought about by regulating proteins involved in growth regulatory pathways and cell cycle [7]. TZDs are also reported to induce G0/G1 arrest and apoptosis of malignant cells by upregulation of the tumor suppressor p53, and control of DNA repair systems and apoptosis [8]. However, the exact mechanism of action and the genes regulated by PPARγ and biological functions of this transcription factor are not known and need elucidation.

Also, due to high levels of toxicity associated with TZDs (e.g. - troglitazone (Rezulin), rosiglitazone (Avandia), and pioglitazone (Actos)), and their recent withdrawal in several countries, there is a need to search for newer PPAR drugs that exhibit better efficacy but lesser toxicity. Phytochemicals in dietary components are increasingly being used as nutritional supplements in treatment of diseases. Due to the plant origin of these supplements they are considered safe for human consumption [9]. Present data reveal that healthy dietary molecules have a pleiotropic role and are able to change cell metabolism from anabolism to catabolism, modulate energy homeostasis and down regulate inflammation by interacting with enzymes, nuclear receptors and transcriptional factors [10]. Towards this end developing and positioning known phytochemicals that bind and activate PPARγ with more efficacy and safety, while promoting health benefits has become an absolute necessity. Also, it is important to identify the dietary molecules able to influence the course of the disease, their targets in the cell, and the molecular mechanisms involved.

Coffee is one of the most widely consumed beverages in the world. The health-promoting properties of coffee are often attributed to its rich phytochemistry, including caffeine, chlorogenic acid, caffeic acid, hydroxyl hydroquinone (HHQ), etc. More recently, coffee consumption has been associated with reductions in the risk of several chronic diseases, including type 2 diabetes mellitus, Parkinson's disease and hepatocellular disease [11-13]. The association between coffee intake and breast cancer risk is biologically plausible because of its complex make-up of chemicals, e.g., caffeine and polyphenolic compounds such as flavonoids and lignans [14-16]. Among them, the relationship between coffee drinking and breast cancer risk holds great interest. Recent meta-analyses demonstrate inverse associations between coffee intake and the risk of colon, liver, breast, and endometrial cancer [17-20]. Also, a high daily intake of coffee has recently been reported to be associated with a statistically significant decrease in ER-negative breast (ER - Estrogen Responsive) cancer among postmenopausal women [21]. A number of previous epidemiologic studies have estimated the association between coffee consumption and breast cancer risk. However, the results are inconsistent [22]. Nevertheless, several reports in literature suggest that coffee consumption reduces the risk of cancer, but the molecular mechanisms of its chemopreventive effects remain unknown. Moreover, the interpretation of these data has often been limited to the role that caffeine plays [23,24].

HHQ is a natural constituent of coffee accounting for main dry matter constituent in roasted beans. Studies exploring the effects of this bioactive compound on mammalian cells are limited. HHQ was observed to dock and form hydrogen bonds with PDB ID - 2PRG (PDB 3-D crystal structure of the Ligand-binding domain of the human peroxisome proliferator activated receptor gamma solved in complexation with Rosiglitazone, the PPAR gamma agonist/ligand). The initial purpose of our investigation is to determine whether HHQ alters the cell viability in estrogen dependent human breast cancer (MCF-7) and estrogen independent (MDA-MB-231) cells as a model system. HHQ was observed to decrease cell viability and colony formation in a dose-responsive manner and ROS was found to significantly increase in HHQ treated cells in a dose-dependent manner in both the cell lines. We examined the involvement of ROS signaling components (ROS levels and membrane potential) and demonstrated that the selective killing of cancer cells is mediated by induction of oxidative stress that leads to apoptosis. These findings were complemented by the finding that caspase-8 is upregulated. Since glucose utilization provides a constant energy supply, as well as precursors for de novo macromolecular biosynthesis, including DNA, RNA, fatty acids and amino acids that are essential for cell growth and proliferation, we further investigated the effect of HHQ on two key glycolytic genes PGK1 and PKM2 (at the ATP generation step) and observed that both the genes are repressed in a dose-dependent manner. These data suggest on the apoptotic and anti-cancer properties of HHQ via PPARγ. Further investigations on these could possibly help us in understanding the molecular mechanisms by which PPARγ regulates disease targets specifically in breast cancer and the use of HHQ in breast cancer therapeutics.

## Results and discussion

Understanding the molecular pathways that link tumor biology to the staggering array of pathologies and genes is of paramount scientific and medical importance. Though, the complexity of the underlying biochemical and molecular mechanisms of breast cancer make metabolic reprogramming and transformation in breast cancer unclear, many dietary compounds have been identified as potential chemopreventive agents. PPARγ is an interesting target for cancer therapy as its expression is elevated in tumors and also because PPARγ activation is reported to result in decreased cell proliferation, decreased G0/G1 to S phase progression, apoptosis and increased terminal differentiation [25-27]. Also, imbalances in expression of target genes forms the core of metabolic syndrome and cancer regulation through atherogenic metabolic triad/lipid triad metabolism modulation by PPARs [28]. Concurrently, increased levels of glycolytic proteins are observed in plasmas of women with breast cancer as a result of upregulation of glycolysis pathway [29].

In this paper, we for the first time report on the use of coffee component HHQ as a potential ligand for PPARγ and its role in induction of apoptosis in breast cancer cells by delineating the glycolytic pathway gene regulation by PPARγ activation.

### Docking

The three-dimensional protein structures can be used to understand ligand binding and to rationally design novel ligands as prospective drug compounds. PPAR agonists typically possess a small polar region and a hydrophobic region that form hydrogen bonds and hydrophobic interactions, respectively, within the ligand binding domain. Several crystal structures of PPARγ in complexation with their ligands are available in the protein data bank (PDB). Here, we used the PDB crystal structure 2PRG (PPARγ with ligand Rosiglitazone) for structure-based identification of HHQ as a potential ligand for PPARγ in breast cancer therapeutics. We also compared the ligand binding properties of the two compounds Rosiglitazone (the known ligand) and HHQ (the proposed novel ligand). The rerank scores for the Rosiglitazone and HHQ were found to be -122.433 and -33.3562, respectively. The hydrogen bond energy values were -5.487 kcal/mol, and -9.460 kcal/mol for Rosiglitazone and HHQ. Rosiglitazone (the ligand in the crystal structure 2PRG) forms 3 hydrogen bonds with the 2PRG (Gln286, His449, Ser289) and HHQ forms 5 hydrogen bonds with 2PRG (Gln286, His449, Tyr473, Ser289, His323). Hydrogen bonding of the ligand to Tyr473 is reported to be the key to the stabilization of the AF-2 region and it has also been shown that [30] agonistic activity of ligands disappears when Tyr473 is mutated. The importance of His323 and His449 has also been reported [31,32]. Our results show that both the ligands have hydrogen bond interactions with key residues - Tyr473 and His 449, thereby providing specificity of interaction that is a fundamental aspect of molecular recognition. The active site residues that interact with HHQ are shown in Table 1 and the hydrogen bonds between each compound and the 2PRG active site are shown in Figure 1.

**Table 1:** Docking results for HHQ and Rosiglitazone.

Drugs	Hydrogen bond score (kcal.mol-1)	Number of hydrogen bonds	Residues of PPARγ binding site interacting with the ligands	Rerank score
HHQ	-9.46033	5	Gln286, His449, Tyr473, Ser289, His323	-33.3562

Rosiglitazone	-5.48771	3	Gln286, His449, Ser289	-122.433


**Figure 1:** **HHQ docked in the ligand binding domain of PPARγ protein crystal structure for PDB solved in conjunction with Rosiglitazone (PDBID: 2PRG)**. **[A] **Represents hydrogen bonds (in black dotted line) observed for Rosiglitazone (in red) with the active site residues in the ligand binding domain of PPARγ (2PRG). **[B] **Represents hydrogen bonds (in black dotted line) observed for HHQ (in yellow) with the active site residues in the ligand binding domain of 2PRG. **[C] **Represents superposition of the best conformation of Rosiglitazone (in red) and HHQ (in yellow) in the ligand binding domain of 2PRG.

### HHQ inhibits cell proliferation and clonogenic survival

To investigate the potential cell growth inhibition of *HHQ*, we first examined the effect of HHQ on cell proliferation and clonogenic survival in human breast adenocarcinomas. For this we chose two breast adenocarcinoma cell lines, MDA-MB-231 (estrogen independent) and MCF-7 (estrogen dependent). MDA-MB-231 and MCF-7 were cultured in the control medium for 24 h, followed by 48 h treatment with different concentrations of HHQ for cytotoxic and anti-proliferative studies. HHQ led to decrease in relative density of viable cells as detected by MTT dye reduction assay. A dose-effect relationship was observed as shown in Figure 2. The IC-50 value for MDA-MB-231 and MCF-7 were found to be 25 μM and 50 μM, respectively. We proceeded with 12.5 μM and 25 μM of HHQ to investigate the comparable effects of same concentration on both the cell lines. At 12.5 μM the relative viability in MDA-MB-231 and MCF-7 was 58.2% and 76.3%, respectively, whereas at 25 μM the relative viability in MDA-MB-231 and MCF-7 was 50% and 60.7%, respectively. As morphological analyses depict the health of a cell, we next examined the cells for any altered morphology on treatment with HHQ. Cells cultured in the presence of HHQ (12.5 μM and 25 μM) show significant morphological changes and were found to be reduced in cell mass as well as number as compared to control. Also, HHQ treatment induced detachment and rounding in breast cancer cells as shown by phase contrast images in both the cell lines (Figure 3 (12.5 μM and 25 μM)). Furthermore, to examine the antitumor activity of HHQ on colony forming potential in breast cancer cells we performed clonogenic assay. This assay is an *in vitro *assay based on the ability of a single cell to proliferate and differentiate into colonies in response to various insults. HHQ severely affected the colony forming potential of human breast cancer cells - MDA-MB-231 and MCF-7. As shown in Figure 4A and 4B clonogenicity of both the breast cancer lines were found to be significantly reduced in a concentration-dependent manner after exposure to HHQ.

**Figure 2:** **Growth curve inhibition as assessed by MTT assay in human breast cancer cells (MDA-MB-231 (blue line) and MCF-7 (grey line))**. The breast cancer cells were exposed to different doses of HHQ for 48 h at 37 °C. The cell viability in breast cancer cells decreased in dose-dependent fashion. The IC-50 value for MDA-MB-231 and MCF-7 were observed to be 25 μM and 50 μM, respectively. Data are representative of three independent experiments done in triplicates and expressed as mean ± S.E.M. *p < 0.005 represents statistical significant difference between control and HHQ test groups.

**Figure 3:** **Phase contrast images of human breast cancer cells (MDA-MB-231 and MCF-7)**. The breast cancer cells were exposed to 12.5 µM and 25 µM concentration of HHQ for 48 h at 37 °C. HHQ treated groups did not retain their normal morphology. HHQ induced cell rounding and detachment in breast cancer cells.

**Figure 4:** **The inhibitory effects of HHQ on colony formation in human breast cancer cells (MDA-MB-231 and MCF-7) as evaluated by clonogenic assay**. The breast cancer cells were exposed to 12.5 µM and 25 µM concentration of HHQ for 48 h at 37 °C. **[A] **Representative plates; **[B] **graph of the number of colonies formed (the result of three independent experiments, expressed as mean ± SEM). Decrease in number of colonies in HHQ treated groups were statistically significant (*P<0.05).

### HHQ induces intracellular ROS generation and cytotoxicity

Reactive oxygen species (ROS) is a universal entity mediating apoptosis [33]. ROS act as a secondary messenger in cell signaling and are essential for various biological processes in normal cells. Disturbances in redox balance relate to human pathogenesis including cancers. ROS are constantly generated and eliminated in the biological system, and play important roles in a variety of normal biochemical functions and abnormal pathological processes. Growing evidence suggests that cancer cells exhibit increased intrinsic ROS stress, due in part to oncogenic stimulation, increased metabolic activity, and mitochondrial malfunction. Since ROS are chemically active and can inflict severe cellular damage, the very fact that cancer cells are under increased intrinsic ROS stress may also provide a unique opportunity to kill the malignant cells based on their vulnerability to further ROS insults caused by exogenous agents [34]. HHQ is earlier reported to generate reactive oxygen species (ROS) by autoxidation [35]. Therefore, to get further insights to HHQ induced cytotoxicity in breast cancer cells; we examined the intracellular ROS generation. As shown in Figure 5, intracellular ROS formation was found to be significantly increased in HHQ treated cells as compared to control cells in a dose-dependent manner. The effective enhancement of ROS production by HHQ correlates to its cytotoxicity nature. Since the mitochondrial respiratory chain (electron transport chain) is a major source of ROS generation in the cells, the vulnerability of the mitochondrial DNA to ROS mediated damage has been suggested to be a mechanism to amplify ROS stress in cancer cells [36]. One major effect is to generate increased intracellular ROS causing loss of outer mitochondrial membrane permeability and induction of apoptosis [37,38]. Another possible mechanism by which cancer cells generate increased amounts of ROS may involve malfunction of the mitochondrial respiratory chain. The fact that cancer cells exhibit an increased dependency on glycolysis to meet their ATP need (the Warburg effect) may reflect an inefficient ATP generation in mitochondria, or "respiration injury" [39]. A correlation between mtDNA mutations and increased ROS contents in primary leukemia cells isolated from patients has been shown [40]. Because the mitochondrial respiratory chain is the major site of ROS generation due to electron transfer, malfunction of the mitochondrial respiratory chain associated with mtDNA mutations is likely to result in more free radical production due to increased "leakage" in mitochondrial membrane.

**Figure 5:** **HHQ induced intracellular ROS production in human breast cancer cells, MDA-MB-231 [A] and MCF-7 [C]**. The breast cancer cells were treated with 12.5 μM and 25 μM of HHQ for 48 h at 37 °C, intracellular ROS was detected by a fluorescent microscope. Quantitation of the ROS signals in MDA-MB-231 and MCF-7 is shown in **[B] **and **[D]**, respectively. Significant increase in ROS level was observed in HHQ treated cells. Data are representative of three independent experiments done in triplicates and expressed as mean ± S.E.M. Increase in ROS generation in HHQ treated groups with 12.5 μM and 25 μM were statistically significant (*P<0.05).

### HHQ induces mitochondrial dysfunctioning

Mitochondria are central players in the determination of cell life and death. Their main physiological function is energy production by the oxidative phosphorylation pathway. This process not only involves production of cell energy currency, ATP but also increases the production of reactive oxygen species (ROS) as by-products of aerobic metabolism. Mitochondria are also the main regulators of apoptotic cell death by mediating extrinsic and intrinsic apoptotic pathways. Oxidative stress may cause oxidative damage to various cellular components and may lead to lipid peroxidation, protein oxidation, mitochondrial DNA mutations, initiation of apoptosis cascade by decrease in mitochondrial membrane potential and release of apoptogenic factor cytochrome c into the cytosol [41]. Thus, the oxidative damage and the associated mitochondrial dysfunction may lead to energy depletion, accumulation of cytotoxic mediators, apoptosis and ultimately cell death. Therefore to investigate the effect of HHQ induced oxidative stress on mitochondria and apoptosis cascade initiation, we undertook mitochondrial membrane potential analysis using potential sensitive, cationic dye JC1. This dye exhibits potential-dependent accumulation in mitochondria, indicated by a fluorescence emission shift from green (525 nm) to red (590 nm). Consequently, live cells have higher red/green intensity ratio as compared to cells undergoing apoptosis. As shown in Figure 6, we observed that the breast cancer cells when treated with HHQ show loss of mitochondria membrane potential (MMP) in a dose-dependent manner. This decrease in MMP at 25 μM of HHQ was significant in both the cell lines. Furthermore, we found that the level of pro-apoptotic protein Bax, significantly increased in a concentration-dependent manner in both the breast cancer cells (Figure 7). The expression levels of Bax correlates with the MMP loss in breast cancer cells on treatment with HHQ. This protein is involved in the mitochondrial apoptotic signaling pathway. The activation of the proapoptotic Bcl-2 family member Bax, induces permeabilization of the mitochondrial outer membrane and release of cytochrome c leading to caspase dependent apoptosis [42,43]. Together, these data corroborate with our previous results and demonstrate that there is disruption in mitochondrial potential, permeability and functioning upon PPARγ activation by HHQ.

**Figure 6:** **HHQ induced loss in mitochondrial membrane potential (MMP) in human breast cancer cells (MDA-MB-231 and MCF-7)**. The breast cancer cells were treated with 12.5 μM and 25 μM of HHQ for 48 h at 37 °C and then immunostained for JC1. HHQ treated cells showed loss of MMP comparable to that of the control cells. Data are representative of three independent experiments done in triplicates and expressed as mean ± S.E.M. *p < 0.005 represents statistical significant difference between control and HHQ test groups.

**Figure 7:** **Expression analyses of pro-apoptotic protein Bax in response to HHQ treatment in human breast cancer cells (MDA-MB-231 and MCF-7)**. The breast cancer cells were treated with 12.5 μM and 25 μM of HHQ for 48 h at 37 °C. Representative western blot hybridization signals of Bax for MDA-MB-231 **[A] **and MCF-7 **[B] **and the quantitation of the signals is shown in **[C] **and **[D]**, respectively. Significant increase in Bax expression was observed in HHQ treated cells. Data are presented as mean ± SEM of three independent experiments. *p< 0.005 represents statistical significant difference between control and HHQ test groups.

### Induction of caspase dependent apoptosis by HHQ

Caspase-8 activation is one of the early events leading to apoptosis. PPAR synthetic ligands are known to activate intrinsic and extrinsic apoptotic cascade [44,45]. In order to understand the mechanism of cell death, we hypothesized that PPARγ ligand HHQ may initiate apoptosis cascade via PPARγ dependent pathway. To examine the above hypothesis we undertook the expression analysis of apoptotic protein, caspase-8. Interestingly, we observed that on treatment with HHQ the level of procaspase-8 decreases significantly in both the cancer cells. This demonstrates that caspase-8 proenzyme is being cleaved to active caspase-8 fragments in a dose-dependent manner (Figure 8). Concurrent increase in proapototic protein Bax, loss of mitochondrial membrane potential and activation of caspase-8 demonstrate PPARγ dependent apoptotic cascade activation by HHQ.

**Figure 8:** **Expression analyses of proenzyme caspase-8 in response to HHQ treatment in human breast cancer cells (MDA-MB-231 and MCF-7)**. The breast cancer cells were treated with 12.5 μM and 25 μM of HHQ for 48 h at 37 °C. Representative western blot hybridization signals for proenzyme caspase-8 for MDA-MB-231 **[A] **and MCF-7 **[B] **and the quantitation of the signals are shown in **[C] **and **[D]**, respectively. Significant decrease in expression of proenzyme caspase-8 was observed in HHQ treated cells. Data are presented as mean ± SEM of three independent experiments. *p< 0.005 represents statistically difference between control and HHQ test groups.

### PPARγ dependent modulation of glycolytic enzymes

In 1930, Otto Warburg discovered the unknown link between highly proliferative nature of cancer cells and glycolysis. The phenomenon involved was described as the "Warburg Effect" which is characterized by increased glucose uptake and dependence on glycolysis for ATP production even in the presence of oxygen source. The glycolytic rate of rapidly proliferating tumor cells was found to be 200 times higher than those of their normal tissues of origin. Altenberg and Greulich (2004) found over expression of glycolytic genes in 24 different types of cancer including breast cancer. Two such glycolytic genes are phosphoglycerate kinase 1 (PGK1) and tumor specific pyruvate kinase muscle 2 (PKM2) [46,47]. PGK1 and PKM2 catalyze the sixth and ninth step, respectively, in the glycolysis pathway generating two ATPs each. PGK1 also functions as a polymerase alpha cofactor protein (primer recognition protein) and is involved in DNA synthesis. PKM2 on the other hand is also a metabolic regulator and is also reported to be involved in channelization of glucose carbons to biosynthetic processes and hence control glycolysis. Hence, down regulating these enzymes would not only starve the cells for ATP but also lead to biosynthetic metabolite starvations, as they are important for tumor cell proliferation and survival. Earlier, we reported that both phosphoglycerate kinase 1 (PGK1) and pyruvate kinase M2 (PKM2) are repressed by PPARγ in the same two breast cancer cell lines MDA-MB-231 and MCF-7. Further analysis suggested that this repression leads to decrease in ATP levels and apoptosis [48]. Here, we hypothesized (based on docking results) that HHQ can modulate the expression of PGK1 and PKM2 via PPARγ dependent pathway. Therefore, to test this hypothesis, we undertook expression analysis of these metabolic enzymes. We observed that the expression of glycolytic genes, PGK1 and PKM2 was significantly reduced in both the breast cancer cells on treatment with HHQ in dose-dependent manner, Figure 9, 10. Further, to confirm the repression of glycolytic genes, PGK1 and PKM2 through HHQ induced PPARγ activation, we utilized GW9662, an irreversible PPARγ antagonist which acts by binding to the human ligand-binding domain (region E/F). As shown in Figure 11, no significant repression of PGK1 and PKM2 was seen on pre-treating the breast cancer cells with GW9662 (10 μM, 4h at 37 °C) followed by HHQ (12.5 μM and 25 μM, 48 h at 37 °C). GW9662 showed no effect of HHQ on expression of PGK1 and PKM2, thereby suggesting that the activation of PPARγ is required for repression of these enzymes. Conversely, these data suggests that HHQ represses the expression of glycolytic enzymes via PPARγ dependent pathway. Down regulation of PGK1 and PKM2 decreases ATP production in the cytoplasm and mitochondria, initiating apoptosis and suppressing cancer metabolism. ATP depletion, used in combination with chemotherapy and/or radiation, has a variety of effects on cancer cells including inducing apoptosis in multi-drug resistant cells and decreasing tumor promotion. Cellular ATP level has been reported as an important determinant of cell death [49]. Though the exact mechanisms of these effects have not been fully elucidated, these investigations suggest on the role of HHQ as an anti-cancer agent. However, further work is required to establish the exact nature and behavior of this molecule in conjunction with other coffee components and to determine its relevance to the biological role of PPARγ breast cancer progression and therapeutics.

**Figure 9:** **Expression analyses of glycolytic enzyme phosphoglycerate kinase 1 (PGK1) in response to HHQ treatment in human breast cancer cells, MDA-MB-231 and MCF-7**. The breast cancer cells were treated with 12.5 μM and 25 μM of HHQ for 48 h at 37 °C. Representative western blot hybridization signals for PGK1 **[A] **and the quantitation of the signals is shown in **[B]**. Immunofluorescent detection of PGK1 is shown in **[C] **and the relative intensity measurement of immunofluorescence is shown in **[D]**. Significant decrease in PGK1 expression was observed in HHQ treated cells. Data are representative of three independent experiments done in triplicates and expressed as mean ± S.E.M. ''*'' represents the statistical significant (p<0.05) difference between control and HHQ treated groups.

**Figure 10:** **Expression analyses of glycolytic enzyme pyruvate kinase-muscle 2 (PKM2) in response to HHQ treatment in human breast cancer cell, MDA-MB-231 and MCF-7**. The breast cancer cells were treated with 12.5 μM and 25 μM of HHQ for 48 h at 37 °C. Representative western blot hybridization signals for PKM2 **[A] **and the quantitation of the signals is shown in **[B]**. Immunofluorescent detection of PKM2 is shown in **[C] **and the relative intensity measurement of immunofluorescence is shown in **[D]**. Significant decrease in PKM2 expression was observed in HHQ treated cells. Data are representative of three independent experiments done in triplicates and expressed as mean ± S.E.M. ''*'' represents the statistical significant (p<0.05) difference between control and HHQ treated groups.

**Figure 11:** **PPARγ dependent repression of glycolytic enzymes PGK1 and PKM2 by HHQ in human breast cancer cells, MDA-MB-231 and MCF-7**. The breast cancer cells were pre-treated with a potent PPARγ antagonist, GW9962 (10 μM) for 4 h at 37 °C, followed by treatment with 12.5 μM and 25 μM of HHQ for 48 h at 37 °C. Representative western blot hybridization signals for PGK1 **[A] **and PKM2 **[B] **for both the breast cancer cell lines and the quantitation of the signals is shown in **[C] **and **[D]**, respectively. GW9662 showed no effect of HHQ on expression of PGK1 and PKM2, thereby suggesting that the activation of PPARγ is required for repression of these enzymes. Data are representative of three independent experiments and expressed as mean ± S.E.M.

## Conclusion

Our results have established previously unknown novel cross-link between HHQ, PPARγ, ROS and glycolysis; thereby adding a new dimension to therapeutic potential of PPARγ ligands. Although the exact mechanism remains unclear and further studies are still needed to clarify the potential role and molecular basis of action of PPARγ in breast carcinogenesis, our investigation open a new direction for development HHQ in breast cancer treatment. Further investigations on these could possibly help us in understanding the molecular mechanisms by which PPARγ regulates disease targets specifically in breast cancer and the use of its ligands in breast cancer therapeutics. Despite several advancements that have been made on the subject, there is still much to be clarified regarding PPARγ signaling in breast cancer and several important questions remain unanswered. Many intriguing avenues of PPARγ research have been opened and hold the potential to ultimately lead to newer classes of more selective molecules.

## Materials and methods

### Docking of HHQ into PPARγ structure

Docking studies were carried out using MolDock™ (Molegro virtual docker) which is based on a new heuristic search algorithm that combines differential evolution with a cavity prediction algorithm (Thomsen & Christensen, 2006). The PDB file for the crystal structure of PPARγ (PDB ID - 2PRG) was downloaded from http://www.rcsb.org and transferred into the workspace keeping the orientation as a control. The energy between the existing ligand and protein was subsequently minimized. Both protein and ligands (Rosiglitazone and HHQ) were optimized in the workspace for docking by the addition of hydrogens. All structural water molecules were removed from the protein molecules using protein preparation wizard. Binding sites in the electrostatic surface of the protein was identified using the grid based cavity prediction algorithm. A total of five cavities were detected and the prepositioned ligand in the active site cavity was identified and the docking was constrained to the predicted active site cavity. MolDock™ scoring function is used for evaluating the energy between the ligand and the protein target. Grid resolution, number of runs, population size, maximum iterations, scaling factor, and cross over rate were set as 0.30 Å, 10, 50, 2000, 0.5, 0.9, respectively, for each run. Multiple poses were returned for each run with the RMSD threshold set to 1.00 Å. The pose with the highest rerank score was retained in the workspace for detailed evaluation of the ligand binding at the active site cavity. MVD was installed in Windows vista operating system on an Intel Core 2.

### Reagents

Dulbecco's modified eagle's medium (1000 mg/L glucose, L-glutamine and sodium bicarbonate), Fetal bovine serum, HHQ, GW9662 and crystal violet were purchased from Sigma-Aldrich (St Louis, MO, USA). Penicillin-Streptomycin-Neomycin antibiotic mixture, Hoechst 33258 and the Image-iTTM LIVE Green Reactive Oxygen Species (ROS) detection reagents were procured from Invitrogen (Eugene, OR, USA) and JC-1dye from Biotium (Hayword, CA, USA). Sodium chloride, Tris base, potassium chloride, sodium di hydrogen phosphate, glycine and sodium phosphate di basic were purchased from Wako Pure Chemical Industries (Osaka, Japan).

### Cell culture and treatments

The human breast adenocarcinoma cell lines MCF-7 and MDA-MB-231 were purchased from the American Type Culture Collection (ATCC; Manassas, VA, USA). The carcinoma cultures were maintained in Dulbecco's modified eagle's medium supplemented with 10% fetal bovine serum and PNS antibiotic mixture 100 ng/ml at 37 °C and 5% CO_2_/95% O_2_. Cultures at about 50% confluency were treated with 12.5 µM and 25 µM of HHQ concentration for 48 h at 37 °C and for PPARγ activity inhibition studies, the breast cancer cells were pre-treated with GW9662 (10 μM, 4h at 37 °C) followed by HHQ (12.5 μM and 25 μM, 48 h at 37 °C) and harvested for further use.

### Cell proliferation assay and morphological study

HHQ was tested for its anti-proliferative activity on MDA-MB-231 and MCF-7 cells using the 3-(4, 5-dimethylthiazol-2-yl)-2, 5-diphenyltetrazolium bromides (MTT) test (Roche, Mannheim, Germany) following manufacturer's instructions. The MTT metabolic activity is a colorimetric cell proliferation assay that identifies living cells, and is based on the cellular conversion of a tetrazolium salt into insoluble formazan, which can be quantified by spectrophotometry. 5 × 10^3 ^cells/ well were plated in 96-well plates and grown for 24 h. The cells were then exposed to varying concentrations of HHQ for 48 h to find the half maximal inhibitory concentration (IC50) values. The intensity of the reduced dye that corresponds to the viable cells was measured at reference wavelength of 570 nm by Thermo Scientific Varioskan Flash Multimode Reader. Morphological changes in breast cancer cells treated with 12.5 µM and 25 µM of HHQ concentration for 48 h were examined by phase contrast microscopy. All experiments were performed in triplicates, and the relative cell viability (%) was expressed as a percentage relative to the untreated control cells.

### Clonogenic assay

Colony formation potential of human breast cancer cells on exposure to HHQ was assessed by clonogenic assay. Clonogenic assay is a cell survival assay based on the ability of a single cell to grow into a colony. To determine long-term effects, breast cancer cells were treated with 12.5 µM and 25 µM of HHQ concentration for 48 h. At the end of treatment the breast cancer cells were then plated at a concentration of 100 cells/well in a new 6-well plate. The cells were allowed to grow for 14 days to form colonies. Fresh medium was replaced every third day. The colonies were washed with PBS and fixed in pre-chilled methanol: acetone mixture (1:1) for 10 min at room temperature. The colonies were then stained with crystal violet dye (0.5% in water) at room temperature for overnight. Cells were washed with water and plates were photographed with image scanner (EPSON GT-1500). Quantitative analysis of the total number of colonies was performed with Image J software (National Institutes of Health).

### Detection of reactive oxygen species

The reactive oxygen species were detected by fluorescent staining using the Image-iTTM LIVE Green Reactive Oxygen Species (ROS) Detection Kit (Molecular Probes Inc, USA). The assay is based on a nonfluorescent and cell permeable 5-(and-6)-carboxy-2',7'-dichlorodihydrofluorescein diacetate (carboxy-H2DCFDA). The carboxy-H2DCFDA permeates the live cells and is deacetylated by intracellular esterases. The reduced fluorescein compound is oxidized by the cellular ROS and emits bright green fluorescence with excitation/ emission maxima of 495/529 nm. The cells were grown on glass cover slips placed in 12-well plate and were treated with 12.5 µM and 25 µM concentration of HHQ for 48 h. Subsequently, cells were fixed and then stained for ROS by following manufacturer's instructions. The images were analyzed with AxioVision software (version 4.4, Carl Zeiss).

### Assessment of mitochondrial membrane potential (ΔΨ)

Mitochondrial transmembrane potential was investigated using a fluorochrome, JC-1 dye (Biotium). JC-1 (5,5',6,6'-tetrachloro-1,1',3,3' tetra ethyl benzimidazolyl carbo cyanine iodide) dye exhibits potential-dependent accumulation of red fluorescent J-aggregates in energized mitochondria. JC-1 exists as a green fluorescent (535 nm) monomer and also accumulates as J-aggregates (595 nm) in the active mitochondria, which stain red. Consequently, healthy cells will exhibit high red/green fluorescence intensity ratio. In apoptotic cells, mitochondrial depolarization is indicated by a decrease in the red/green fluorescence intensity ratio. Therefore this fluorescence emission shift from green (~529 nm) to red (~590 nm) is indicative of mitochondrial depolarization occurring during apoptosis. After 48 h of 12.5 µM and 25 µM of HHQ treatment, the cells were incubated with 1X JC-1 dye at 37 °C for 15 min followed by washes with assay buffer. The red fluorescence (excitation 550 nm, emission 600 nm) and green fluorescence (excitation 485 nm, emission 535 nm) were measured using fluorescence Thermo Scientific Varioskan Flash Multimode plate reader. The ratio of red fluorescence to green fluorescence was determined in JC-1 stained cells. The relative mitochondrial membrane potential (%) was expressed as a percentage relative to the untreated control cells.

### Immunocytostaining

In order to find out the modulation of test proteins by HHQ through PPARγ, the test protein were immunostained. For immunostaining, cells were plated on glass coverslips in a 12-well plate (10^4 ^cells/coverslip). The cells were allowed to attach for 24 h and then exposed to 12.5 µM and 25 µM of HHQ for 48 h. At the end of treatment cells were washed with cold PBS three times and then fixed with pre-chilled methanol: acetone mixture (1:1) for 10 min at room temperature. Fixed cells were washed twice with PBS, permeabilized with 0.32% Triton X-100 in PBS (PBST) for 10 min and blocked with 2% bovine serum albumin (BSA) in PBS for 30 min. The cells were then probed with anti-PGK1 (1:250; Abcam, Cambridge, UK), anti-PKM2 (1:250; Abcam, Cambridge, UK), antibodies for overnight at 4°C. After primary antibody incubation the cells were washed thrice with 0.1% PBST, and then incubated with secondary antibodies (Alexa-594-conjugated goat anti-rabbit and Alexa 488-conjugated goat anti-mouse, (Molecular Probes, Eugene, OR) for 1 h at room temperature followed by 3 times washing with 0.1% PBST and then once with PBS. The coverslips were then mounted with ProLong+® Gold antifade reagent (Molecular Probes, Inc.) and observed under a microscope (Axiovert 200M; Carl Zeiss, Thornwood, NY). The experiment was carried out in duplicate in three independent experiments. The images were analyzed with Axio Vision software (version 4.4, Carl Zeiss).

### Western blot analysis

Expression level of indicated proteins was examined by Western blotting. The control and treated cells were lysed in RIPA lysis buffer (25 mM Tris-HCl (pH 7.6), 1% NP-40, 1% sodium deoxycholate, 150 mM NaCl, 0.1% SDS) complemented with complete protease inhibitors (Roche) for 15 min on ice followed by centrifugation at 14,000 *g *for 15 min at 4 °C. The protein concentration was determined using BCA reagents (Pierce, Rockford, IL, USA). Protein lysate (20 µg) was resolved in 10% in SDS-polyacrylamide gel under standard denaturing conditions according to Laemmli's method (1970) followed by transfer onto polyvinylidene difluoride membranes using a Trans-Blot SD (Bio-Rad, Lewes, E. Sussex, UK.) semi-dry electroblotter for 30 min at 20 V. Subsequently, the membranes were blocked for 45 min at room temperature with 2% bovine serum albumin in 0.1% PBST. The membranes were then probed with anti-PGK1 (1:1000; Abcam, Cambridge, UK), anti-PKM2 (1:500, Abcam), anti-caspase-8 (1:1000; Cell Signaling, Boston, MA, USA), Anti-Bax (1:1000; Cell Signaling) and anti-β-actin (1:20,000; Abcam) at 4°C overnight followed by three washes for 5 min each with 0.1% PBST. The membranes were then incubated with horseradish peroxidase conjugated secondary antibody (1:20,000; Abcam) for 45 min at RT and washed thrice for 5 min each with 0.1% PBST followed by chemiluminescent detection using Luminescent Image Analyzer equipped with charge-coupled device camera (LAS-4000 Ver. 2.1; Fuji Film, Tokyo, Japan).

### Data analysis

The captured images for ROS assay and immunostaining were analyzed using AxioVision software (version 4.4; Carl Zeiss). The analysis determined the overall density of ROS, PGK1 and PKM2 immunoreactivity in 5-8 randomly selected fields in each slide. The mean intensity of ROS, PGK1, and PKM2 immunoreactivity in control and treated cells were evaluated and presented as a histogram. Similarly the Relative Optical Density (%) for immunoreactive bands in western blotting for PGK1, PKM2 and Caspase-8 were analyzed using Image J software (National Institutes of Health).

### Statistical analysis

The quantitative data are representative of three independent experiments done in triplicates and expressed as mean ± SEM. Statistical analysis was performed using analysis of variance (one way analysis of variance) followed by Bonferroni's on test to determine differences in mean and *p *< 0.05 was considered as statistically significant.

## Competing interests

The authors declare that they have no conflict of interest.

## Authors' contributions

MKS, YN designed the project. SKD and KRS carried out computational analysis. BS, KS and RS performed the experiments. MKS, KRS and BS analyzed the results and wrote the manuscript. All authors read and approved the final manuscript.

## Declarations

Publication of this article was funded by University of Tsukuba, Japan.

This article has been published as part of *BMC Genomics *Volume 14 Supplement 5, 2013: Twelfth International Conference on Bioinformatics (InCoB2013): Computational biology. The full contents of the supplement are available online at http://www.biomedcentral.com/bmcgenomics/supplements/14/S5.
